The article "Weighted single-step GWAS identified candidate genes associated with semen traits in a Duroc boar population" was published in 2019. Journal: BMC Genomics.

# Weighted single-step GWAS identified candidate genes associated with semen traits in a Duroc boar population

**DOI:** 10.1186/s12864-019-6164-5

**Published:** 2019-10-30

**Authors:** Ning Gao, Yilong Chen, Xiaohong Liu, Yunxiang Zhao, Lin Zhu, Ali Liu, Wei Jiang, Xing Peng, Conglin Zhang, Zhenshuang Tang, Xinyun Li, Yaosheng Chen

**Affiliations:** 1 State Key Laboratory of Biocontrol, School of Life Sciences, Sun Yat-Sen University, North Third Road, Guangzhou Higher Education Mega Center, Guangzhou, 510006 China; 2 Key Laboratory of Agricultural Animal Genetics, Breeding, and Reproduction of the Ministry of Education, Huazhong Agricultural University, Wuhan, 430070 China; 3 Guangxi Xiubo genetics technology Co., LTD, Guigang, 537100 China; 4 Guangxi Yangxiang Agriculture and Husbandry Co., LTD, Guigang, 537100 China

**Keywords:** Candidate genes, Duroc pigs, Semen traits, Sperm motility, Weighted single-step GWAS

## Abstract

**Background:**

In the pig production industry, artificial insemination (AI) plays an important role in enlarging the beneficial impact of elite boars. Understanding the genetic architecture and detecting genetic markers associated with semen traits can help in improving genetic selection for such traits and accelerate genetic progress. In this study, we utilized a weighted single-step genome-wide association study (wssGWAS) procedure to detect genetic regions and further candidate genes associated with semen traits in a Duroc boar population. Overall, the full pedigree consists of 5284 pigs (12 generations), of which 2693 boars have semen data (143,113 ejaculations) and 1733 pigs were genotyped with 50 K single nucleotide polymorphism (SNP) array.

**Results:**

Results show that the most significant genetic regions (0.4 Mb windows) explained approximately 2%~ 6% of the total genetic variances for the studied traits. Totally, the identified significant windows (windows explaining more than 1% of total genetic variances) explained 28.29, 35.31, 41.98, and 20.60% of genetic variances (not phenotypic variance) for number of sperm cells, sperm motility, sperm progressive motility, and total morphological abnormalities, respectively. Several genes that have been previously reported to be associated with mammal spermiogenesis, testes functioning, and male fertility were detected and treated as candidate genes for the traits of interest: Number of sperm cells, *TDRD5*, *QSOX1*, *BLK*, *TIMP3*, *THRA*, *CSF3*, and *ZPBP1*; Sperm motility, *PPP2R2B*, *NEK2*, *NDRG*, *ADAM7*, *SKP2*, and *RNASET2*; Sperm progressive motility, *SH2B1*, *BLK*, *LAMB1*, *VPS4A*, *SPAG9*, *LCN2, and DNM1*; Total morphological abnormalities, *GHR*, *SELENOP*, *SLC16A5*, *SLC9A3R1*, and *DNAI2*.

**Conclusions:**

In conclusion, candidate genes associated with Duroc boars’ semen traits, including the number of sperm cells, sperm motility, sperm progressive motility, and total morphological abnormalities, were identified using wssGWAS. KEGG and GO enrichment analysis indicate that the identified candidate genes were enriched in biological processes and functional terms may be involved into spermiogenesis, testes functioning, and male fertility.

## Background

In the pig production industry, artificial insemination (AI) plays an important role in enlarging the beneficial impact of elite boars. Sperm quality, affected by genetic and environmental factors simultaneously and with moderate to low heritability [1, 2], is essential for guaranteeing the success of AI. For both academic researchers and AI station managers, understanding the genetic background and detecting genetic markers associated with semen traits can help in improving genetic selection for such traits and accelerate genetic progress. Biologically, the process of spermatogenesis, which mainly contains three steps including mitotic phase, meiotic phase, and spermiogenesis, involves complex coordination among many genes and different cell types and occurs in the seminiferous tubules of the testes [3]. Mutations in related genes and status changes in corresponding cells will potentially affect the sperm quality and male fertility. From the aspect of genetic control and animal breeding, detecting candidate genes responsible to sperm quality and fertility is an essential step.

With the fast development of sequencing technology and commercially availability of dense marker panels, researchers can precisely identify quantitative trait loci (QTL) by searching for association between genetic markers and phenotypic records, which is known as genome-wide association study (GWAS) [4]. Though many challenges, such as the need for efficient study design especially for replication efforts and technologies for capturing genetic variation, the missing heritability problem, reducing the bias introduced into a dataset, and utilizing of new resources available, remained to be addressed [5], GWAS has been successfully implemented in detecting genetic risk factors for human diseases and mapping QTL for economically important traits in both animal and plant breeding populations. Among the established GWAS approaches, the weighted single step GWAS (wssGWAS) [6] is preferable for association study in domesticated animals, for which large numbers of individuals are usually phenotyped but less genotyped. Technically, the wssGWAS calculates genomic estimated breeding values (GEBVs) of individuals by solving mixed model equations using **H** (a blend of pedigree derived relationship matrix **A** and weighted genomic relationship matrix **G**_***w***_**,** which is constructed in the manner of weighting SNPs according to their genetic variances, [7, 8]) as relatedness matrix, and converts the GEBVs into marker effects in the genotyped subpopulation based on the underlying equivalency between marker effect models and breeding value models. Genetic variance of certain chromosome window is subsequently calculated as the variation of the genetic values possessed by SNPs located in that window (i.e., *Var*(**Z**_*window*_**g**_*window*_), **Z**_*window*_ and **g**_*window*_ represent genotypes and marker effects of SNPs located in the window, respectively).

In several previous studies related to boar semen traits, associated genetic markers or candidate genes have been reported for both sperm quantity (i.e. number of sperm cells per ejaculation) and quality (i.e. sperm motility and morphological abnormalities) traits, [9–13]. However, the genetic background of breeds or boar populations, number of boars used for association study, and density of genetic marker panels varied a lot among the previous studies. The Duroc boars have been used as terminal sire in most of the modern three-way crossbreeding pig production system. While due to the relatively small numbers of Duroc boars in one herd and difficulty in phenotypic data collecting, seldom association studies have been conducted. In this study, we utilized wssGWAS to detect genetic regions and further candidate genes associated with semen traits in a Duroc boar population. In order to further understand the genetic control of semen traits, post GWAS analyses, KEGG and GO enrichment were performed to find biological processes and functional terms in which the candidate genes were involved.

## Results

In this study, we identified genomic regions associated with semen traits in a Duroc boar population via wssGWAS [6]. In order to investigate the genetic background of the semen traits under consideration, we estimated the heritabilities of these traits by fitting model (1) using the pedigree derived numerator relationship matrix. Variance component and heritability estimations are presented in Table 1. The estimated heritabilities were 0.18, 0.16, 0.16, and 0.26 for the number of sperm cells, sperm motility, sperm progressive motility, and total morphological abnormalities, respectively. The heritability ranged from moderate to low, which were at the similar magnitude compared to Marques et al., (2018, 2017) while higher than that of Wolf (2010), in which relatively smaller Large White and Landrace boar populations were used for heritability estimation.

**Table 1:** Variance component and heritability estimates of semen traits

Traits^a^	Vg	Vpe	Ve	h^2^(SE)
lnNcells	0.05172	0.03682	0.19380	0.18320 (0.01687)
MOT	0.00069	0.00062	0.00299	0.16019 (0.02070)
PMOT	0.00757	0.00248	0.03695	0.16105 (0.01092)
ABN	0.00170	0.00105	0.00376	0.26134 (0.02744)

^a^*lnNcells* Number of sperm cells, *MOT* Motility, *PMOT* Progressive motility, *ABN* Total morphological abnormalities

Figure 1 shows the proportion of variances explained by each 0.4 Mb windows for the traits under study. Table 2 shows the first three most important QTL regions and the candidate genes, which have been previously reported to be associated with mammal spermiogenesis, testes functioning, and male fertility, for the four traits. Overall, the first three QTL regions together explained about 5.12~11.97% of the genetic variances of the semen traits under study (Table 2). For each trait, the most important windows explained approximately 2%~ 6% of the total genetic variances (Table 2). Furthermore, the identified windows (windows that explained more than 1% of total genetic variances) explained totally 28.29, 35.31, 41.98, and 20.60% of genetic variances (not phenotypic variance) for number of sperm cells, sperm motility, sperm progressive motility, and total morphological abnormalities, respectively (Fig. 1 and Additional file 1: Table S1, Additional file 2: Table S2, Additional file 3: Table S3 and Additional file 4: Table S4). From the aspect of pig breeding, the relatively high proportions of genetic variances explained by the identified QTL regions may imply the possibility of integrating these QTL mapping results into estimating of genetic breeding values of semen traits [14, 15].

**Fig. 1:** Proportion of genetic variances of the semen traits explained by 0.4 Mb windows. lnNcells: number of sperm cells; **MOT:** motility; **PMOT:** Progressive motility; **ABN:** Total morphological abnormalities

**Table 2:** First three most important QTL regions and candidate genes for semen traits

Traits^a^	chr	Position (Mb)	nSNPs	gVar(%)	Candidate genes
lnNcells	9	121.15–121.95	8	3.79	TDRD5, QSOX1
	14	14.49–15.29	16	2.26	BLK
	5	11.71–12.51	8	2.14	TIMP3
MOT	13	1.29–2.09	5	4.51	–
	2	147.71–148.51	12	3.08	PPP2R2B
	9	131.55–132.35	13	2.58	NEK2
PMOT	15	135.89–136.69	10	5.81	–
	7	0.13–0.93	16	3.82	–
	4	5.15–5.95	17	2.34	–
ABN	13	1.25–2.05	7	1.93	–
	16	26.76–27.56	7	1.76	GHR, SELENOP
	12	6.20–7.00	9	1.43	SLC16A5, SLC9A3R1, DNAI2

^a^ *lnNcells* Number of sperm cells, *MOT* Motility, *PMOT* Progressive motility, *ABN* Total morphological abnormalities. Within each trait, genomic regions were decreasingly sorted based on the proportion of genetic variance explained

Table 3 shows the GO terms and KEGG pathways in which the identified genes enriched. Four GO terms and one KEGG pathway were enriched for the number of sperm cells. The enriched GO terms are involved in *positive regulation of myeloid cell differentiation* (GO:0045639), *steroid hormone mediated signaling pathway* (GO:0043401), *granulocyte colony-stimulating factor receptor binding* (GO:0005130), and *enzyme regulator activity* (GO:0030234). The enriched KEGG pathway is involved in *thyroid hormone signaling* (ssc04919). For sperm motility, three GO terms were enriched for the candidate genes, while no KEGG pathway was targeted. The GO terms play roles in *cellular calcium ion homeostasis* (GO:0006874), *protein phosphorylation* (GO:0006468), and *protein kinase activity* (GO:0004672). For progressive motility, seven GO terms and two KEGG pathways were enriched for the identified candidate genes. These GO terms and KEGG pathways are involved in nucleotide metabolic and biosynthesis processes. Three GO terms were enriched for the total morphological abnormalities, while no KEGG pathway was targeted. These GO terms are related to *transition between slow and fast fiber* (GO:0014886), *sensory perception of sound* (GO:0007605), *endochondral ossification* (GO:0001958), *cullin family protein binding* (GO:0097602), *RNA polymerase II transcription factor activity,* and *sequence-specific DNA binding* (GO:0000981).

**Table 3:** GO terms and KEGG pathways where the candidate genes significantly (*p* < 0.05) enriched

Traits^a^	Term^b^	Count	Genes	*P*-Value
lnNcells	GO:0045639~positive regulation of myeloid cell differentiation	2	CSF3	0.017295
	GO:0043401~steroid hormone mediated signaling pathway	2	THRA, NR1D1	0.045478
	GO:0005130~granulocyte colony-stimulating factor receptor binding	2	CSF3	0.006326
	GO:0030234~enzyme regulator activity	2	PSMD3, MTMR9	0.034316
	ssc04919:Thyroid hormone signaling pathway	3	THRA, GATA4, MED24	0.040606
MOT	GO:0006874~cellular calcium ion homeostasis	3	SLC24A4, ATP2C1, SLC30A1	0.010583
	GO:0006468~protein phosphorylation	3	ST3GAL1, NEK2, PIK3R4	0.027143
	GO:0004672~protein kinase activity	3	NEK2, MAP3K14, PIK3R4	0.041698
PMOT	GO:0006163~purine nucleotide metabolic process	3	NME2, NME1, ADSL	0.000208
	GO:0006220~pyrimidine nucleotide metabolic process	2	NME2, NME1	0.026186
	GO:0006241~CTP biosynthetic process	2	NME2, NME1	0.029872
	GO:0009142~nucleoside triphosphate biosynthetic process	2	NME2, NME1	0.029872
	GO:0006228~UTP biosynthetic process	2	NME2, NME1	0.029872
	GO:0006183~GTP biosynthetic process	2	NME2, NME1	0.037203
	GO:0044822~poly(A) RNA binding	7	TUFM, ATXN2L, UTP18, NME1, NIP7, SNTB2, DNM1	0.04506
	ssc01100:Metabolic pathways	10	ST6GALNAC6, NME2, PIP5KL1, PTGES2, ST6GALNAC4, GMDS, NME1, ADSL, DPM2, FDFT1	0.039824
	ssc01130:Biosynthesis of antibiotics	4	NME2, NME1, ADSL, FDFT1	0.043421
ABN	GO:0014886~transition between slow and fast fiber	2	GTF2I, GTF2IRD1	0.004569
	GO:0007605~sensory perception of sound	3	USH1G, RPL38, SLC9A3R1	0.008744
	GO:0001958~endochondral ossification	2	IMPAD1, PEX7	0.035996

^a^ *lnNcells* Number of sperm cells, *MOT* Motility, *PMOT* Progressive motility, *ABN* Total morphological abnormalities. Within each trait, genomic regions were decreasingly sorted based on the proportion of genetic variance explained

^b^ *GO* Gene Ontology, *KEGG*, Kyoto Encyclopedia of Genes and Genomes pathway

## Discussion

In this study, we conducted association study for boar semen traits in a large Duroc population. To our knowledge, this is the first time that genome-wide association study results are reported in such a large Duroc boar population. Based on the literature (cited above), some of the identified candidate genes have been previously reported to be involved in mammal spermiogenesis, testes functioning, and male fertility. Among the candidate genes identified in this study, *DNAI2* was previously reported to be associated with sperm motility of large white boars [9], while no more genes overlapped with that identified in large white and landrace boars. Similarly, in the study conducted by Marques et al., [9], where wssGWAS was also used, no overlapping regions were identified between large white and landrace boars. However, gene network analysis revealed that genes identified in different lines were involved in the same biological processes [9]. Therefore, it is hard to draw the conclusion that the identified candidate genes in this study are specific to Duroc line. Nevertheness, functional validation experiments of homologous genes in human and model organisms (literature mentioned in the following paragraphs) in the literature provided evidence of role of the identified genes in semen traits. Considering genetic improvement of semen traits, the identified candidate genes may provide knowledge for developing genomic prediction models based on the trait-specific genomic best linear unbiased prediction (GBLUP) [15] by assigning higher genetic variances to genetic markers located in these regions.

For number of sperm cells, 18 relevant QTL regions located on SSC2 (SSC: *Sus scrofa* chromosome), 3, 5, 9, 10, 12, 14, 15, 16, and 17 were identified. Sixty-five genes were annotated in these genomic regions according to the National Center for Biotechnology Information (NCBI) (Additional file 1: Table S1). Among the identified genes, some has been previously reported to be associated with sperm biological function. The *Tudor domain-containing protein 5* (*TDRD5*) and *quiescin Q6/sulfhydryl oxidase 1* (*QSOX1*), located in the region of 121.15–121.95 Mb on SSC9, were considered as candidate gene for the number of sperm cells (Table 2). *TDRDs* are an evolutionarily conserved family of proteins involved in germ cell development, and *TDRD5* is required for retrotransposon silencing, chromatoid body assembly, and spermiogenesis in mice [16]. The *QSOX* family was reported to have biological functions in male germ cell development [17]. BLK gene, located in the region of 14.49–15.29 Mb on SSC14, is an Src-related tyrosine kinase in the events leading to proper sperm formation. Previous study reported that BLK is involved in sperm function and integrity [18]. The members of *tissue inhibitor of metalloproteinase* (*TIMP*), among which *TIMP3* was identified in the region of 11.71–12.51 Mb on SSC5, were reported to exist in human seminal plasma as complexes and may play roles in sperm function [19]. The *thyroid hormone receptor alpha* (*THRA*), identified in the region of 22.19–22.56 Mb on SSC12, is responsible for sertoli cell development, sperm production, and testis weight [20] by regulating the function of triiodothyronine (T3), which played a key role in Sertoli cell development [21]. *Colony stimulating factor 3* (*CSF3*), another gene located in the region of 22.19–22.56 Mb on SSC12, is involved in reactive oxygen species (ROS) of sperm cells and associated with abnormalities in sperm histone transition [22]. A third gene located in the region of 22.19–22.56 Mb on SSC12, *Zona pellucida binding protein 1* (*ZPBP1*), a spermatid and spermatozoon protein, is responsible for sperm morphology. Lin et al., (2007) reported that male mice lacking *ZPBP1* were sterile, with abnormal round-headed sperm morphology and no forward sperm motility.

For sperm motility, 20 relevant QTL regions located on SSC1, 2, 3, 4, 7, 8, 9, 12, 13, 14, 15, 16, and 17 were identified. Fifty-nine genes were annotated in these genomic regions (Additional file 2: Table S2). Within the window explained the largest proportion of genetic variance of sperm motility (1.29–2.09 Mb on SSC13), six genes were targeted, while none of them have ever been previously reported to be associated with semen traits. The protein *phosphatase 2 regulatory subunit B beta* gene (*PPP2R2B*), located in the region of 147.71–148.51 Mb on SSC2, was indicated to be associated with biology of sperm in a Co-Expression Network Analysis conducted in *Bos taurus* and *Sus scrofa* [23]. For the *NIMA related kinase 2* (*NEK2*) gene, located in the region of 131.55–132.35 Mb on SSC9 and showed biased expression in reproductive tissues (testis of human and ovary of swine), several studies have demonstrated its role in the process of meiotic cell cycle and the first meiotic division in mouse spermatocytes [24–27]. *Ndrp3*, a member of the N-myc downstream regulated gene family (*NDRG*), is enhanced expressed specifically in germ cells and involved in regulation of the male meiosis in mouse [18]. The ADAM metallopeptidase domain 7 (*ADAM7*), which located in the region of 8.49–8.86 Mb on SSC14, is associated with epididymosomes, integrated into sperm plasma membrane, and related to fertility and sperm integrity [28, 29]. S-phase kinase associated protein 2 (*SKP2*) was identified in the region of 21.48–21.86 Mb on SSC16. The *Skp2* protein is the receptor subunit of an SCF-type ubiquitin ligase and is a major regulator of the progression of cells into S phase of the cell cycle, *Skp2*-deficient mice shown reduction in the number of mature gametes and thus decreased fertility [30]. Moreover, *Skp2* was reported to be involved in the manipulation of boar sperm production [31]. The ribonuclease T2 (*RNASET2*) gene, located in the region of 1.77–2.16 Mb on SSC1, have been reported to be involved in sperm motility impairment [32] and interacted with *AKAP4* in human sperm tail and subsequently reduced sperm motility by suppressing PKA/PI3K/calcium signaling pathways [33].

For progressive motility, 24 relevant QTL regions located on SSC1, 2, 3, 4, 5, 6, 7, 8, 9, 10, 11, 12, 13, 14, 15, 16, and 17 were identified (Additional file 3: Table S3). Seventy-three genes were annotated in these regions. Within the first three genomic regions that explained the largest proportions of genetic variance, 11 genes were identified but none of them have been previously reported to be directly associated with semen traits in the literatures. However, in the region of 18.51–18.87 Mb on SSC3, SH2B adaptor protein 1 (*SH2B1*) was identified. Previous study in mice have shown that expression of *Sh2b1* on the mRNA level in obesity mice was decreased, which resulted in significant reduction in male fertility and exacerbated reproductive toxicity and germ cell mutagenicity [34]. Src family tyrosine kinase (*BLK*), also identified for the number of sperm cells, is an Src-related tyrosine kinases in the events leading to proper sperm formation, was reported to potentially involved in sperm function and integrity [18]. Laminin subunit beta 1 (*LAMB1*) gene, which directs the expression of beta-galactosidase during development of the mouse testis and ovary [35], was identified in the region of 107.72–108.07 Mb on SSC9. Acuolar protein sorting 4 homolog A (*VPS4A*) gene, located in the region of 17.44–17.8 Mb on SSC6, was previously reported to be involved in human sperm acrosome reaction [36]. Sperm associated antigen 9 (*SPAG9*) gene, which codes an acrosomal molecule that plays role in acrosome reaction and sperm-egg binding [37], was identified in the region of 27.39–27.78 Mb on SSC12. Lipocalin 2 (*LCN2*) gene, located in the region of 268.37–268.73 Mb on SSC1, is involved in sperm maturation and fertilization [38]. Dynamin 1 (*DNM1*), another gene located in the same region on SSC1, acts as a key mediator of sperm acrosome formation and function, is essential for mammalian spermatogenesis [39].

For total morphological abnormalities, 16 relevant QTL regions located on SSC1, 3, 4, 8, 9, 10, 11, 12, 13, 15, 16, and 17 were identified (Additional file 4: Table S4). Sixty-seven genes were annotated in these regions according to NCBI. The *growth hormone receptor* (*GHR*) gene, which shows significant association with embryos survival rate and involved in fertilization rate of dairy cattle [40], was identified in the region of 26.76–27.56 Mb on SSC16 (Table 2). Selenoprotein P (*SELENOP*), another gene located in the same region, is abundantly expressed in the testis and affected the sperm quality of rats [41]. Solute carrier family 16 member 5 (*SLC16A5*) gene, for which a protein-coding variation is associated with cisplatin-induced ototoxic effects and involved in human germ cell testicular cancer [42], was identified in the region of 6.20–7.00 Mb on SSC12. SLC9A3 regulator 1 (*SLC9A3R1*), another gene located in the same region, is important for mouse sperm capacitation through functional interactions with *SLC26A3*, *SLC26A6*, and *CFTR* [43]. Dynein axonemal intermediate chain 2 (*DNAI2*) gene, of which mutations may resulted in defects of sperm flagella in human [9, 44, 45], was identified on SSC12.

## Conclusions

In conclusion, we identified candidate genes associated with the number of sperm cells, sperm motility, sperm progressive motility, and total morphological abnormalities in a Duroc boar population using wssGWAS. Functional validation experiments of homologous genes in human and model organisms (literature mentioned in the Discussion section) in the literature provided evidence of role of the identified genes in semen traits. The identified candidate genes may provide knowledge for developing genomic evaluation models by assigning higher weights to genetic markers located in these regions.

## Methods

### Phenotypes, genotypes, and pedigree

The studied Duroc boar population was a mixed herd consisted of boars from pure Danish lines, pure American lines, and progenies from the crosses between Danish and American Duroc lines. For more detailed description of the conditions where the boars were raised, please refer to our recently published paper [46]. Overall, 5284 pigs (12 generations) were included in the pedigree, of which 2693 boars with semen trait records. Four traits, total sperm morphological abnormalities (ABN), number of sperm cells (Ncells), sperm motility (MOT, defined as proportion of moving sperms), and sperm progressive motility (PMOT, defined as proportion of sperms moving in strait line) were recorded in the years from 2015 to 2018. The fresh semen was evaluated immediately after ejaculate using the UltiMateTM CASA system (Hamilton Thorne Inc., Beverly, MA, USA). Number of sperm cells was calculated as the product of the semen volume (mL) and concentration (10^6^ mL^− 1^). For the traits of total morphological abnormalities, number of sperm cells, and motility, 143,113 individual ejaculates (53 ejaculates per boar on average) of 2693 boars were used for the association study (Table 4). For the trait progressive motility, 29,526 observations of 1304 out of the 2693 boars were used for association study (Table 4).

**Table 4:** Descriptive statistics of semen traits in the Duroc boar population

Traits^a^	#obs.	#indiv	Min	Median	Mean	Max	SD	CV (%)
lnNcell	143,113	2693	20.70	27.26	27.20	29.37	0.51	1.88
MOT	143,113	2693	0.50	0.90	0.89	1.00	0.07	7.46
PMOT	29,526	1304	0.00	0.57	0.54	0.91	0.15	27.11
ABN	143,113	2693	0.00	0.10	0.12	0.60	0.08	65.94

^a^*lnNcells* Number of sperm cells, *MOT* Motility, *PMOT* Progressive motility, *ABN* Total morphological abnormalities, *#obs*. Number of observations, *#indiv* Number of boars

Total DNA of 1733 pigs were extracted (semen of boars and ear tissue samples of sows) using the genome extraction kits produced by Wuhan NanoMagBio Technology Co., Ltd. Those pigs were genotyped using the GGP 50 k SNP array (GeneSeek, US), which contains 50,703 SNPs. Overall, 1627 out of the genotyped pigs were related to boars with phenotypic records through pedigree and used for further analysis. SNPs, for which the Sscrofa10.2 physical positions were provided by the SNP array producer, were remapped to Sscrofa11.1 using the genome remapping procedure available in NCBI (https://www.ncbi.nlm.nih.gov/). SNPs with unknown positions (9405 SNPs) and that unable to map to Sscrofa11.1 (1842 SNPs) were removed from the dataset. Moreover, SNPs on sex chromosomes (2469 SNPs) were excluded to avoid sex bias in constructing genomic relationship matrix and calculating genetic breeding values (1231 boars and 392 sows were included in the genotype file and used for constructing the genomic relationship matrix). Autosome SNPs were filtered via plink [47] using the following criteria: individual call rate ≥90% (4 pigs removed); SNP call rate ≥90% (673 SNPs removed); minor allele frequency ≥0.01 (5345 SNPs removed); Hardy–Weinberg equilibrium *p*-value ≥10^−6^ (2680 SNPs removed). After quality control, 1623 pigs, among which 1231 had semen evaluation data, and 28,289 SNPs remained for further analysis. Missing genotypes were finally imputed using Beagle software (version 4.1) [48, 49].

### Statistical model

The weighted single step GWAS procedure [6, 50] was used for association study. Briefly, genomic estimated breeding values (GEBVs) were estimated via a weighted single step GBLUP and marker effects were calculated from the GEBVs. QTL regions were selected based on the proportion of genetic variance explained by certain chromosome segments.

The following repeatability model was used in this study.

1 $$ \mathbf{y}=\mathbf{Xb}+\mathbf{Za}+\mathbf{Wp}+ Age+ Intv+\mathbf{e},\kern1.25em $$

where **y** denoted the response; **X**, **Z**, and **W** denoted the design matrices; **b** was fixed effects (overall mean and year-season of ejaculation); $\mathbf{a}\sim \mathrm{N}\left(0,\mathbf{H}{\sigma}_a^2\right)$ was a vector of genetic values; $\mathbf{p}\sim \mathrm{N}\left(0,\mathbf{I}{\sigma}_p^2\right)$ was a vector of random permanent boar effect; covariates *Age* and *Intv* denoted the age of the boars at months when ejaculating and collection interval (days), respectively. $\mathbf{e}\sim \mathrm{N}\left(0,\mathbf{I}{\sigma}_e^2\right)$ denoted the residuals. **I** denoted the identity matrix. The inverse of **H** matrix, a blend of pedigree and genetic marker derived matrices [7, 8], was calculated as

$$ {\mathbf{H}}^{-1}={\boldsymbol{A}}^{-1}+\left[\begin{array}{cc}\mathbf{0}& \mathbf{0}\\ {}\mathbf{0}& {\boldsymbol{G}}_{\omega}^{-1}-{\boldsymbol{A}}_{22}^{-1}\end{array}\right], $$

where ***A*** denoted the pedigree derived relationship matrix; ***A***_22_ was a sub matrix of ***A*** corresponding to the genotyped individuals; ***G***_*ω*_ **=** 0.9***G*** + 0.1***A***_22_, these weights were used to scale the genomic information to be compatible with the pedigree information and to control bias [51, 52]; $\boldsymbol{G}=\frac{\boldsymbol{Z}\boldsymbol{D}{\boldsymbol{Z}}^{\prime }}{\sum_{i=1}^m2{p}_i\left(1-{p}_i\right)}$ was the genomic relationship matrix [53], where ***Z*** was a matrix of genotypes (with 0-2p, 1-2p, and 2-2p represented genotypes AA, Aa, and aa, respectively; p denoted the minor allele frequency (MAF)), ***D*** denoted a diagonal matrix contained the SNP weights, *p*_*i*_ denoted MAF of the *i*^*th*^ SNP, and *m* denoted the number of SNPs.

Variance components and further heritability of the studied traits were obtained via average information restricted maximum likelihood (AI-REML) [54] procedure using pedigree. Marker effects and further weights for constructing ***G*** were calculated in an iterative way used by Wang et al., [6, 50]. An iteration procedure with the following steps was used for association study.

- Step1: Initialization, let t = 1, ***D***_(*t*)_ **=** ***I***, ***G***_(*t*)_ **=** λ***ZD***_(*t*)_***Z***^′^, and $\uplambda =\frac{1}{\sum_{i=1}^m2{p}_i\left(1-{p}_i\right)}$;
- Step2: GEBV estimation, calculate GEBVs ($\hat{\boldsymbol{a}}$) via ssGBLUP with $$ {\mathbf{H}}^{-1}={\boldsymbol{A}}^{-1}+\left[\begin{array}{cc}\mathbf{0}& \mathbf{0}\\ {}\mathbf{0}& {\left(0.9{\boldsymbol{G}}_{(t)}+0.1{\boldsymbol{A}}_{22}\right)}^{-\mathbf{1}}-{\boldsymbol{A}}_{22}^{-1}\end{array}\right] $$;
- Step3: Marker effects calculation, obtain marker effects via ${\hat{\boldsymbol{g}}}_{(t)}=\uplambda {\boldsymbol{D}}_{(t)}{\boldsymbol{Z}}^{\prime }{\boldsymbol{G}}_{(t)}^{-1}\hat{\boldsymbol{a}}$;
- Step4: SNP weights calculation, get SNP weights for the next iteration via ${d}_{i\left(t+1\right)}={\hat{g}}_{i(t)}^22{p}_i\left(1-{p}_i\right)$;
- Step5: SNP weights normalization, rescale the weights to keep the total genetic variance constant via ${\boldsymbol{D}}_{\left(t+1\right)}=\frac{tr\left({\boldsymbol{D}}_{(1)}\right)}{tr\left({\boldsymbol{D}}_{\left(t+1\right)}\right)}{\boldsymbol{D}}_{\left(t+1\right)}$;
- Step 6: Weighted ***G*** construction, calculate ***G*** for the next iteration via ***G***_(*t* + 1)_ **=** λ***ZD***_(*t* + 1)_***Z***^′^;
- Step7: Let *t* = *t* + 1 and loop to step 2.

The procedure was run for three iterations, as used in Wang et al., [50] and Marques et al., [9], and marker effects obtained from the third iteration were used for calculating proportions of genetic variances explained by subsets of consecutive SNPs. SNPs located within 0.4 Mb (average haploblock length of the commercial pig lines including Duroc [55]) of unoverlapping windows were grouped into subsets and the genetic variances explained by those windows were obtained via

$$ \frac{Var\left({\boldsymbol{a}}_i\right)}{\sigma_a^2}\times 100\%=\frac{Var\left({\sum}_{j=1}^M{\boldsymbol{Z}}_j{g}_j\right)}{\sigma_a^2}\times 100\%. $$

The iteration steps mentioned above were run with BLUF90 software families [51] in a iterative way, AIREMLF90 for variance components estimation, BLUPF90 for GEBVs calculation, and postGSf90 [56] for marker effects converting, respectively.

### Candidate genes detection and functional enrichment analysis

QTL regions were selected according to genetic variance of chromosome windows. Windows explained higher than 1% genetic variances were selected as candidate QTL regions, within which candidate genes were searched. The threshold of 1% was set based on literature [9, 57–59] and the expected average genetic variance explained by single chromosome segment (0.027, 100% divided by 3707 windows). Consecutive windows with midpoints less than 0.4 Mb apart were treated as overlapped and merged. The first three windows that explained the largest amount of genetic variances were further extended to 0.4 Mb flanking regions of the midpoints on both upstream and downstream.

Candidate genes on “National Center for Biotechnology Information” (NCBI, http://www.ncbi.nlm.nih.gov) were searched in the selected QTL regions. Kyoto Encyclopedia of Genes and Genomes (KEGG) [60] and Gene Ontology (GO) [61] enrichment analyses were performed based on candidate gens for each trait via the Database for Annotation, Visualization, and Integrated Discovery (DAVID, Version 6.8, https://david.ncifcrf.gov/) [62].

## Supplementary information

**Additional file 1: Table S1.** Genomic regions explained more than 1% of genetic variance for the number of sperm cells.

**Additional file 2: Table S2.** Genomic regions explained more than 1% of genetic variance for sperm motility.

**Additional file 3: Table S3.** Genomic regions explained more than 1% of genetic variance for progressive motility.

**Additional file 4: Table S4.** Genomic regions explained more than 1% of genetic variance for total morphological abnormalities.

## Data Availability

The datasets generated and/or analyzed during the current study are not publicly available since the studied population is consisted of the nucleus herd of Guangxi Yangxiang Agriculture and Husbandry Co.,LTD, but are available from the corresponding author on reasonable request.

## Abbreviations

ABN: Total sperm morphological abnormalities
AI: Artificial insemination
AI-REML: Average information restricted maximum likelihood
Co., Ltd.: Company limited
DAVID: The database for annotation, visualization, and Integrated discovery
GBLUP: Genomic best linear unbiased prediction
GEBVs: Genomic estimated breeding values
GO: Gene ontology
KEGG: Kyoto Encyclopedia of Genes and Genomes
MAF: Minor allele frequency
MOT: Sperm motility
NCBI: National Center for Biotechnology Information
Ncells: Number of sperm cells
PMOT: Sperm progressive motility
QTL: Quantitative trait loci
SNP: Single nucleotide polymorphism
SSC: *Sus scrofa* chromosome
SYSU: Sun Yat-Sen University
wssGWAS: Weighted single-step GWAS
